# 2,2′-Dimethyl-7,7′-(methyl­enediimino)di-1,8-naphthyridin-1-ium bis­(perchlorate)

This article has been retracted.

**DOI:** 10.1107/S1600536808024616

**Published:** 2008-08-06

**Authors:** Juan Mo, Jian-Hua Liu, Yu-Shan Pan, Su-Mei Zhang, Xiang-Dang Du

**Affiliations:** a College of Animal Husbandry and Veterinary Studies, Henan Agricultural University, Zhengzhou, Henan Province 450002, People’s Republic of China

## Abstract

In the title salt, C_19_H_20_N_6_^2+^·2ClO_4_^−^, the two planar 1,8-naphthyridine systems are linked by a methyl­enediamine group with a dihedral angle of 60.6 (1)° between the two systems. The crystal structure involves extensive N—H⋯O and C—H⋯O hydrogen bonding.

## Related literature

For related literature, see: Baker & Norman (2004 ▶); Gavrilova & Bosnich (2004 ▶); Nakatani *et al.* (2000 ▶, 2001 ▶); Stadie *et al.* (2007 ▶); Ferrarini *et al.* (1997 ▶).

## Experimental

### 

#### Crystal data

C_19_H_20_N_6_^2+^·2ClO_4_^−^
*M* *_r_* = 531.31
Orthorhombic,
*a* = 8.191 (1) Å
*b* = 19.325 (2) Å
*c* = 27.885 (2) Å
*V* = 4413.9 (5) Å^3^
*Z* = 8
Mo *K*α radiation
μ = 0.36 mm^−1^
*T* = 113 (2) K
0.34 × 0.16 × 0.14 mm

#### Data collection

Bruker SMART CCD area-detector diffractometer
Absorption correction: multi-scan (*SADABS*; Sheldrick, 1996 ▶) *T*_min_ = 0.908, *T*_max_ = 0.952
31220 measured reflections
3882 independent reflections
3598 reflections with *I* > 2σ(*I*)
*R*_int_ = 0.061

#### Refinement

*R*[*F* ^2^ > 2σ(*F* ^2^)] = 0.060
*wR*(*F* ^2^) = 0.134
*S* = 1.16
3882 reflections
308 parameters
16 restraints
H atoms treated by a mixture of independent and constrained refinement
Δρ_max_ = 0.35 e Å^−3^
Δρ_min_ = −0.41 e Å^−3^

### 

Data collection: *SMART* (Bruker, 1997 ▶); cell refinement: *SAINT* (Bruker, 1997 ▶); data reduction: *SAINT*; program(s) used to solve structure: *SHELXS97* (Sheldrick, 2008 ▶); program(s) used to refine structure: *SHELXL97* (Sheldrick, 2008 ▶); molecular graphics: *XP* in *SHELXTL* (Sheldrick, 2008 ▶); software used to prepare material for publication: *XP* in *SHELXTL*.

## Supplementary Material

Crystal structure: contains datablocks global, I. DOI: 10.1107/S1600536808024616/hg2415sup1.cif

Structure factors: contains datablocks I. DOI: 10.1107/S1600536808024616/hg2415Isup2.hkl

Additional supplementary materials:  crystallographic information; 3D view; checkCIF report

## Figures and Tables

**Table 1:** Hydrogen-bond geometry (Å, °)

*D*—H⋯*A*	*D*—H	H⋯*A*	*D*⋯*A*	*D*—H⋯*A*
N1—H1⋯O6^i^	0.88 (4)	1.92	2.794 (4)	168
N3—H3*A*⋯O3	0.80 (3)	2.23	2.990 (6)	159
N4—H4*A*⋯O5^i^	0.71 (4)	2.56	3.233 (5)	160
N4—H4*A*⋯O7^i^	0.71 (4)	2.52	3.133 (5)	145
N6—H6⋯O1	0.84 (3)	2.00	2.838 (8)	178
C1—H1*A*⋯O7^ii^	0.98	2.54	3.501 (3)	167
C1—H1*B*⋯O4^iii^	0.98	2.33	3.078 (4)	132
C4—H4⋯O8^iv^	0.95	2.52	3.392 (7)	152
C10—H10*B*⋯O4^iv^	0.99	2.35	3.082 (5)	130
C13—H13⋯O2^i^	0.95	2.41	3.259 (3)	149
C19—H19*B*⋯O5	0.98	2.57	3.351 (6)	136
C19—H19*C*⋯O7^v^	0.98	2.58	3.207 (7)	122
C19—H19*C*⋯O8^v^	0.98	2.57	3.548 (4)	172

Symmetry codes: (i) ; (ii) ; (iii) ; (iv) ; (v) .

## supplementary crystallographic information

### Comment

1,8-Naphthyridine and its derivatives are used for binding of mismatched guanine or used as versatile ligands which are able to form metal aggregates with monodentates fashion or chelating bidentate fashion(Nakatani *et al.*, 2000; Nakatani *et al.*, 2001; Ferrarini *et al.*, 1997; Gavrilova & Bosnich, 2004; Baker & Norman, 2004; Stadie *et al.*, 2007). We report here a new 1,8-Naphthyridine compound (Fig. 1).

The title compound reveals 1,8-naphthyridine rings are linked by methenediamine with a dihedral angle between two 1,8-naphthyridine rings of 60.6 (1)°. Each 1,8-naphthyridine ring is an almost planar in which the ten atoms forming the 1,8-naphthyridine ring have mean deviation of 0.03Å from the least-squares plane calculated using the ten atoms. To balance hydrogen ion charge of two 1,8-naphthyridine rings, there are two perchlorate groups in crystal cell. From the packing diagram (Fig. 2), it seems that the intramolecular N–H···O and C–H···O and hydrogen bonds are effective in the stabilization of the crystal structure.

### Experimental

To the solution of 2-amino-7-methyl-1,8-naphthyridine (3.18 g, 0.02 mol) in mixed solvent of water (28 mL) and ethanol (2 mL), 37% formadehyde solution (0.86 mL, 0.01 mol) was added dropwise at 0°C and the reaction mixture was stirred at room temperature for 24h. The white precipitate formed was filtered, washed several times with water and then with diethyl ether and dried. Yield: 55% (1.81 g). FTIR (KBr)cm^-1^: ν_NH_ 3389, 3266; ν_CH_ 3026. Anal. Calc. For C_19_H_18_N_6_: C, 69.07; H, 5.49; N, 25.44. Found: C, 68.86; H, 5.56; N, 25.37. Single crystals of (I) suitable for an X-ray study were obtained by slow evaporation of an aqueous ethanol solution (30% *v*/*v*) under the conditions in the presence of perchloric acid at 293 K over a period of one month.

### Refinement

Hydrogen atoms of NH (naphthyridine and amine) were located in a Fourier map and refined freely. All the other hydrogen atoms were generated geometrically (C—H bond lengths of methyl group fixed at 0.98Å, C—H bond lengths of naphthyridine fixed at 0.95 Å) assigned appropriated isotropic thermal parameters, *U*_iso_(H) = 1.2*U*_eq_(C). Each perchlorate anion is disordered over two different orientations. The Cl–O distances were restrained to 1.43 (4)Å.

### Crystal data

**Table:**

C_19_H_20_N_6_^2+^·2ClO_4_^–^	*F*_000_ = 2192
*M**_r_* = 531.31	*D*_x_ = 1.599 Mg m^−^^3^
Orthorhombic, *P**b**c**a*	Mo *K*α radiation λ = 0.71070 Å
Hall symbol: -P 2ac 2ab	Cell parameters from 7263 reflections
*a* = 8.1910 (5) Å	θ = 2.1–28.0º
*b* = 19.3250 (12) Å	µ = 0.36 mm^−^^1^
*c* = 27.8850 (19) Å	*T* = 113 (2) K
*V* = 4413.9 (5) Å^3^	Prism, colorless
*Z* = 8	0.34 × 0.16 × 0.14 mm

### Data collection

**Table:**

Bruker SMART CCD area-detector diffractometer	3882 independent reflections
Radiation source: fine-focus sealed tube	3598 reflections with *I* > 2σ(*I*)
Monochromator: graphite	*R*_int_ = 0.061
Detector resolution: 7.31 pixels mm^-1^	θ_max_ = 25.0º
*T* = 113(2) K	θ_min_ = 2.1º
φ and ω scans	*h* = −9→9
Absorption correction: multi-scan(SADABS; Sheldrick, 1996)	*k* = −22→22
*T*_min_ = 0.909, *T*_max_ = 0.952	*l* = −33→32
31220 measured reflections	

### Refinement

**Table:**

Refinement on *F*^2^	Secondary atom site location: difference Fourier map
Least-squares matrix: full	Hydrogen site location: inferred from neighbouring sites
*R*[*F*^2^ > 2σ(*F*^2^)] = 0.060	H atoms treated by a mixture of independent and constrained refinement
*wR*(*F*^2^) = 0.134	*w* = 1/[σ^2^(*F*_o_^2^) + (0.0498*P*)^2^ + 5.3196*P*] where *P* = (*F*_o_^2^ + 2*F*_c_^2^)/3
*S* = 1.16	(Δ/σ)_max_ = 0.003
3882 reflections	Δρ_max_ = 0.35 e Å^−^^3^
308 parameters	Δρ_min_ = −0.41 e Å^−^^3^
16 restraints	Extinction correction: none
Primary atom site location: structure-invariant direct methods	

### Special details

**Table:**

Geometry. All e.s.d.'s (except the e.s.d. in the dihedral angle between two l.s. planes) are estimated using the full covariance matrix. The cell e.s.d.'s are taken into account individually in the estimation of e.s.d.'s in distances, angles and torsion angles; correlations between e.s.d.'s in cell parameters are only used when they are defined by crystal symmetry. An approximate (isotropic) treatment of cell e.s.d.'s is used for estimating e.s.d.'s involving l.s. planes.
Refinement. Refinement of *F*^2^ against ALL reflections. The weighted *R*-factor *wR* and goodness of fit *S* are based on *F*^2^, conventional *R*-factors *R* are based on *F*, with *F* set to zero for negative *F*^2^. The threshold expression of *F*^2^ > σ(*F*^2^) is used only for calculating *R*-factors(gt) *etc*. and is not relevant to the choice of reflections for refinement. *R*-factors based on *F*^2^ are statistically about twice as large as those based on *F*, and *R*- factors based on ALL data will be even larger.

### Fractional atomic coordinates and isotropic or equivalent isotropic displacement parameters (Å^2^)

**Table:**

	*x*	*y*	*z*	*U*_iso_*/*U*_eq_	Occ. (<1)
Cl1	0.24246 (10)	0.22574 (4)	0.56855 (3)	0.0360 (2)	
Cl2	1.00163 (9)	0.01682 (3)	0.69459 (3)	0.0323 (2)	
O1	0.1693 (6)	0.1730 (2)	0.59780 (16)	0.0534 (14)	0.747 (5)
O2	0.3894 (5)	0.2014 (2)	0.5483 (2)	0.0758 (17)	0.747 (5)
O3	0.1302 (6)	0.2438 (2)	0.53084 (12)	0.0738 (15)	0.747 (5)
O4	0.2651 (6)	0.28664 (19)	0.59698 (15)	0.0700 (14)	0.747 (5)
O5	0.8509 (4)	0.02894 (17)	0.67091 (14)	0.0664 (12)	0.870 (6)
O6	0.9850 (5)	−0.03196 (14)	0.73264 (10)	0.0657 (13)	0.870 (6)
O7	1.1129 (3)	−0.01123 (15)	0.65972 (10)	0.0490 (10)	0.870 (6)
O8	1.0661 (6)	0.0802 (2)	0.7134 (2)	0.0444 (13)	0.870 (6)
O1'	0.1358 (14)	0.1676 (5)	0.5766 (4)	0.039 (3)	0.253 (5)
O2'	0.3710 (11)	0.2233 (6)	0.6037 (3)	0.062 (4)	0.253 (5)
O3'	0.3135 (14)	0.2178 (6)	0.5220 (3)	0.062 (4)	0.253 (5)
O4'	0.1558 (13)	0.2875 (4)	0.5708 (4)	0.052 (3)	0.253 (5)
O5'	0.8301 (12)	0.0031 (10)	0.7058 (7)	0.053 (6)	0.130 (6)
O6'	1.0870 (19)	−0.0453 (6)	0.7069 (7)	0.048 (6)	0.130 (6)
O7'	1.012 (3)	0.0307 (10)	0.6446 (4)	0.062 (7)	0.130 (6)
O8'	1.056 (3)	0.0738 (10)	0.7228 (8)	0.039 (10)	0.130 (6)
N1	0.1466 (3)	0.16498 (13)	0.27420 (9)	0.0328 (6)	
N2	0.1460 (3)	0.16453 (12)	0.35633 (8)	0.0293 (6)	
N3	0.1396 (3)	0.16601 (15)	0.43819 (10)	0.0353 (6)	
N6	0.3295 (3)	0.04505 (14)	0.58097 (9)	0.0336 (6)	
N5	0.2041 (3)	0.04253 (13)	0.50731 (9)	0.0327 (6)	
N4	0.0922 (4)	0.04231 (16)	0.43264 (11)	0.0417 (7)	
C2	0.1739 (4)	0.19127 (16)	0.23034 (10)	0.0377 (8)	
C3	0.2463 (5)	0.25570 (18)	0.22665 (11)	0.0435 (9)	
H3	0.2634	0.2759	0.1960	0.052*	
C4	0.2935 (4)	0.29061 (16)	0.26746 (11)	0.0390 (8)	
H4	0.3453	0.3344	0.2647	0.047*	
C5	0.2662 (4)	0.26239 (14)	0.31277 (10)	0.0285 (7)	
C6	0.1858 (4)	0.19774 (14)	0.31595 (10)	0.0268 (6)	
C7	0.1866 (4)	0.19636 (15)	0.39716 (10)	0.0288 (7)	
C8	0.2786 (4)	0.25928 (15)	0.39855 (10)	0.0314 (7)	
H8	0.3132	0.2779	0.4284	0.038*	
C9	0.3159 (4)	0.29193 (15)	0.35722 (10)	0.0324 (7)	
H9	0.3748	0.3343	0.3578	0.039*	
C1	0.1243 (6)	0.14783 (18)	0.18868 (12)	0.0518 (10)	
H1A	0.2123	0.1154	0.1808	0.078*	
H1B	0.1026	0.1776	0.1610	0.078*	
H1C	0.0253	0.1219	0.1968	0.078*	
C16	0.4320 (4)	0.02351 (16)	0.61578 (11)	0.0360 (8)	
C17	0.5112 (4)	−0.03943 (17)	0.60916 (12)	0.0402 (8)	
H17	0.5862	−0.0556	0.6326	0.048*	
C18	0.4812 (4)	−0.07835 (17)	0.56878 (12)	0.0398 (8)	
H18	0.5322	−0.1222	0.5653	0.048*	
C14	0.3773 (4)	−0.05443 (15)	0.53293 (12)	0.0357 (7)	
C15	0.3015 (4)	0.01043 (16)	0.53928 (11)	0.0316 (7)	
C11	0.1802 (4)	0.00934 (17)	0.46592 (11)	0.0368 (8)	
C12	0.2463 (4)	−0.05808 (16)	0.45608 (12)	0.0424 (8)	
H12	0.2221	−0.0808	0.4267	0.051*	
C13	0.3428 (4)	−0.08878 (16)	0.48880 (12)	0.0411 (8)	
H13	0.3878	−0.1332	0.4825	0.049*	
C19	0.4554 (5)	0.06921 (19)	0.65809 (11)	0.0446 (8)	
H19A	0.4863	0.1156	0.6473	0.067*	
H19B	0.5418	0.0503	0.6785	0.067*	
H19C	0.3533	0.0718	0.6763	0.067*	
C10	0.0224 (4)	0.10976 (18)	0.43970 (12)	0.0431 (8)	
H10A	−0.0336	0.1106	0.4712	0.052*	
H10B	−0.0612	0.1178	0.4147	0.052*	
H3A	0.163 (4)	0.1865 (17)	0.4619 (12)	0.035 (10)*	
H1	0.101 (5)	0.124 (2)	0.2764 (13)	0.055 (11)*	
H4A	0.081 (5)	0.0269 (19)	0.4097 (13)	0.040 (12)*	
H6	0.281 (4)	0.0828 (18)	0.5853 (12)	0.035 (9)*	

### Atomic displacement parameters (Å^2^)

**Table:**

	*U*^11^	*U*^22^	*U*^33^	*U*^12^	*U*^13^	*U*^23^
Cl1	0.0433 (5)	0.0317 (4)	0.0331 (4)	−0.0003 (3)	0.0046 (4)	−0.0008 (3)
Cl2	0.0360 (5)	0.0256 (4)	0.0353 (4)	−0.0007 (3)	0.0018 (3)	−0.0012 (3)
O1	0.064 (3)	0.046 (2)	0.050 (3)	0.016 (2)	0.026 (2)	0.022 (2)
O2	0.055 (3)	0.049 (2)	0.124 (4)	−0.002 (2)	0.053 (3)	−0.011 (3)
O3	0.118 (4)	0.059 (2)	0.045 (2)	0.031 (2)	−0.025 (2)	0.0033 (18)
O4	0.089 (3)	0.052 (2)	0.070 (3)	−0.001 (2)	0.002 (3)	−0.027 (2)
O5	0.0421 (19)	0.063 (2)	0.095 (3)	0.0139 (15)	−0.0291 (19)	−0.019 (2)
O6	0.126 (4)	0.0396 (16)	0.0313 (15)	−0.0408 (19)	−0.0042 (19)	0.0050 (12)
O7	0.0410 (17)	0.0542 (18)	0.0519 (18)	−0.0075 (14)	0.0127 (14)	−0.0213 (14)
O8	0.055 (3)	0.0232 (18)	0.055 (2)	−0.0038 (16)	−0.002 (2)	−0.0076 (17)
O1'	0.036 (6)	0.030 (5)	0.051 (7)	−0.003 (4)	0.014 (5)	0.002 (5)
O2'	0.049 (6)	0.086 (7)	0.052 (6)	−0.022 (5)	−0.013 (5)	0.031 (5)
O3'	0.056 (7)	0.087 (7)	0.041 (6)	−0.016 (6)	0.023 (5)	−0.020 (5)
O4'	0.063 (6)	0.027 (4)	0.065 (6)	0.017 (4)	0.012 (5)	0.007 (4)
O5'	0.030 (8)	0.067 (9)	0.061 (10)	0.008 (7)	0.004 (7)	0.003 (8)
O6'	0.046 (9)	0.033 (8)	0.064 (10)	0.009 (7)	0.000 (8)	0.003 (7)
O7'	0.085 (11)	0.060 (10)	0.041 (9)	−0.012 (8)	0.014 (8)	−0.003 (7)
O8'	0.053 (14)	0.032 (13)	0.032 (12)	0.002 (8)	−0.006 (8)	−0.010 (8)
N1	0.0448 (17)	0.0233 (13)	0.0302 (14)	−0.0046 (12)	−0.0070 (12)	0.0000 (10)
N2	0.0321 (14)	0.0275 (12)	0.0283 (13)	−0.0027 (11)	−0.0009 (11)	0.0035 (10)
N3	0.0381 (16)	0.0419 (15)	0.0260 (14)	0.0023 (13)	−0.0004 (12)	0.0032 (12)
N6	0.0353 (15)	0.0344 (15)	0.0310 (14)	0.0059 (13)	0.0054 (12)	0.0103 (12)
N5	0.0314 (14)	0.0360 (14)	0.0306 (13)	−0.0023 (11)	0.0053 (11)	0.0101 (11)
N4	0.0479 (19)	0.0467 (18)	0.0306 (16)	−0.0128 (14)	−0.0024 (15)	0.0084 (14)
C2	0.053 (2)	0.0331 (16)	0.0266 (16)	0.0011 (15)	−0.0066 (15)	−0.0008 (13)
C3	0.064 (2)	0.0381 (18)	0.0287 (16)	−0.0036 (17)	−0.0008 (16)	0.0063 (14)
C4	0.050 (2)	0.0317 (16)	0.0349 (17)	−0.0098 (15)	0.0017 (15)	0.0043 (13)
C5	0.0341 (17)	0.0212 (14)	0.0302 (15)	−0.0031 (12)	−0.0020 (13)	−0.0004 (12)
C6	0.0325 (16)	0.0223 (13)	0.0257 (14)	−0.0012 (12)	−0.0021 (13)	−0.0003 (11)
C7	0.0299 (16)	0.0301 (15)	0.0264 (15)	0.0067 (13)	0.0012 (13)	0.0022 (12)
C8	0.0359 (18)	0.0293 (15)	0.0290 (15)	0.0050 (13)	−0.0035 (13)	−0.0066 (12)
C9	0.0374 (18)	0.0262 (15)	0.0335 (16)	−0.0018 (13)	−0.0029 (14)	−0.0030 (12)
C1	0.083 (3)	0.0408 (19)	0.0316 (18)	−0.0031 (19)	−0.0128 (19)	−0.0052 (15)
C16	0.0290 (17)	0.0429 (18)	0.0362 (17)	−0.0019 (14)	0.0067 (14)	0.0172 (14)
C17	0.0313 (18)	0.0449 (19)	0.0444 (19)	0.0015 (15)	0.0056 (15)	0.0222 (16)
C18	0.0337 (18)	0.0324 (17)	0.053 (2)	0.0026 (14)	0.0174 (16)	0.0202 (15)
C14	0.0355 (18)	0.0285 (15)	0.0430 (18)	−0.0041 (14)	0.0150 (15)	0.0115 (14)
C15	0.0287 (17)	0.0350 (16)	0.0309 (16)	−0.0028 (13)	0.0097 (13)	0.0104 (13)
C11	0.0381 (19)	0.0409 (18)	0.0314 (16)	−0.0138 (15)	0.0053 (15)	0.0099 (14)
C12	0.052 (2)	0.0331 (17)	0.0417 (19)	−0.0172 (16)	0.0116 (17)	0.0006 (15)
C13	0.048 (2)	0.0273 (16)	0.048 (2)	−0.0080 (15)	0.0165 (17)	0.0061 (14)
C19	0.042 (2)	0.058 (2)	0.0341 (17)	−0.0008 (17)	0.0011 (16)	0.0121 (16)
C10	0.0343 (19)	0.061 (2)	0.0343 (18)	−0.0038 (17)	0.0030 (15)	0.0176 (16)

### Geometric parameters (Å, °)

**Table:**

Cl1—O4'	1.390 (7)	C2—C3	1.383 (5)
Cl1—O2	1.410 (4)	C2—C1	1.490 (4)
Cl1—O3'	1.430 (7)	C3—C4	1.378 (4)
Cl1—O4	1.431 (3)	C3—H3	0.9500
Cl1—O1	1.436 (4)	C4—C5	1.394 (4)
Cl1—O2'	1.439 (7)	C4—H4	0.9500
Cl1—O3	1.440 (3)	C5—C6	1.415 (4)
Cl1—O1'	1.441 (8)	C5—C9	1.424 (4)
Cl2—O5	1.420 (3)	C7—C8	1.431 (4)
Cl2—O7'	1.423 (9)	C8—C9	1.349 (4)
Cl2—O8'	1.424 (10)	C8—H8	0.9500
Cl2—O6	1.426 (3)	C9—H9	0.9500
Cl2—O6'	1.432 (9)	C1—H1A	0.9800
Cl2—O8	1.433 (3)	C1—H1B	0.9800
Cl2—O7	1.439 (3)	C1—H1C	0.9800
Cl2—O5'	1.464 (9)	C16—C17	1.390 (5)
N1—C2	1.343 (4)	C16—C19	1.486 (5)
N1—C6	1.364 (4)	C17—C18	1.376 (5)
N1—H1	0.88 (4)	C17—H17	0.9500
N2—C7	1.336 (4)	C18—C14	1.392 (5)
N2—C6	1.336 (4)	C18—H18	0.9500
N3—C7	1.342 (4)	C14—C15	1.410 (4)
N3—C10	1.451 (4)	C14—C13	1.427 (5)
N3—H3A	0.80 (3)	C11—C12	1.437 (5)
N6—C16	1.350 (4)	C12—C13	1.345 (5)
N6—C15	1.360 (4)	C12—H12	0.9500
N6—H6	0.84 (3)	C13—H13	0.9500
N5—C11	1.335 (4)	C19—H19A	0.9800
N5—C15	1.348 (4)	C19—H19B	0.9800
N4—C11	1.337 (4)	C19—H19C	0.9800
N4—C10	1.437 (5)	C10—H10A	0.9900
N4—H4A	0.71 (4)	C10—H10B	0.9900
			
O4'—Cl1—O2	137.8 (4)	N1—C2—C3	118.7 (3)
O4'—Cl1—O3'	109.9 (6)	N1—C2—C1	116.8 (3)
O4'—Cl1—O4	48.3 (4)	C3—C2—C1	124.5 (3)
O2—Cl1—O4	112.7 (3)	C4—C3—C2	120.0 (3)
O3'—Cl1—O4	122.6 (5)	C4—C3—H3	120.0
O4'—Cl1—O1	111.8 (5)	C2—C3—H3	120.0
O2—Cl1—O1	110.3 (3)	C3—C4—C5	120.8 (3)
O3'—Cl1—O1	127.5 (5)	C3—C4—H4	119.6
O4—Cl1—O1	108.9 (3)	C5—C4—H4	119.6
O4'—Cl1—O2'	111.7 (6)	C4—C5—C6	118.5 (3)
O2—Cl1—O2'	68.8 (5)	C4—C5—C9	125.9 (3)
O3'—Cl1—O2'	108.5 (6)	C6—C5—C9	115.6 (3)
O4—Cl1—O2'	63.6 (5)	N2—C6—N1	116.0 (2)
O1—Cl1—O2'	84.0 (4)	N2—C6—C5	126.2 (3)
O4'—Cl1—O3	59.9 (5)	N1—C6—C5	117.8 (3)
O2—Cl1—O3	109.5 (3)	N2—C7—N3	117.0 (3)
O3'—Cl1—O3	67.9 (5)	N2—C7—C8	123.0 (3)
O4—Cl1—O3	106.7 (2)	N3—C7—C8	120.0 (3)
O1—Cl1—O3	108.7 (3)	C9—C8—C7	119.6 (3)
O2'—Cl1—O3	166.5 (4)	C9—C8—H8	120.2
O4'—Cl1—O1'	110.7 (6)	C7—C8—H8	120.2
O2—Cl1—O1'	108.6 (6)	C8—C9—C5	119.4 (3)
O3'—Cl1—O1'	107.7 (6)	C8—C9—H9	120.3
O4—Cl1—O1'	129.3 (5)	C5—C9—H9	120.3
O2'—Cl1—O1'	108.2 (6)	C2—C1—H1A	109.5
O3—Cl1—O1'	85.2 (5)	C2—C1—H1B	109.5
O5—Cl2—O7'	64.3 (8)	H1A—C1—H1B	109.5
O5—Cl2—O8'	113.6 (11)	C2—C1—H1C	109.5
O7'—Cl2—O8'	112.1 (10)	H1A—C1—H1C	109.5
O5—Cl2—O6	111.8 (2)	H1B—C1—H1C	109.5
O7'—Cl2—O6	149.3 (8)	N6—C16—C17	117.7 (3)
O8'—Cl2—O6	97.5 (11)	N6—C16—C19	117.9 (3)
O5—Cl2—O6'	132.4 (7)	C17—C16—C19	124.4 (3)
O7'—Cl2—O6'	111.3 (8)	C18—C17—C16	120.2 (3)
O8'—Cl2—O6'	111.4 (10)	C18—C17—H17	119.9
O6—Cl2—O6'	46.6 (7)	C16—C17—H17	119.9
O5—Cl2—O8	110.5 (2)	C17—C18—C14	121.0 (3)
O7'—Cl2—O8	100.1 (8)	C17—C18—H18	119.5
O6—Cl2—O8	109.1 (3)	C14—C18—H18	119.5
O6'—Cl2—O8	116.7 (8)	C18—C14—C15	118.3 (3)
O5—Cl2—O7	107.38 (19)	C18—C14—C13	125.9 (3)
O7'—Cl2—O7	50.9 (8)	C15—C14—C13	115.8 (3)
O8'—Cl2—O7	117.9 (11)	N5—C15—N6	116.0 (3)
O6—Cl2—O7	108.3 (2)	N5—C15—C14	125.9 (3)
O6'—Cl2—O7	62.4 (8)	N6—C15—C14	118.1 (3)
O8—Cl2—O7	109.6 (3)	N5—C11—N4	116.8 (3)
O5—Cl2—O5'	45.2 (7)	N5—C11—C12	123.1 (3)
O7'—Cl2—O5'	107.7 (8)	N4—C11—C12	120.2 (3)
O8'—Cl2—O5'	108.7 (10)	C13—C12—C11	119.5 (3)
O6—Cl2—O5'	68.2 (8)	C13—C12—H12	120.3
O6'—Cl2—O5'	105.3 (8)	C11—C12—H12	120.3
O8—Cl2—O5'	115.5 (8)	C12—C13—C14	119.8 (3)
O7—Cl2—O5'	133.2 (8)	C12—C13—H13	120.1
C2—N1—C6	124.2 (3)	C14—C13—H13	120.1
C2—N1—H1	118 (2)	C16—C19—H19A	109.5
C6—N1—H1	117 (2)	C16—C19—H19B	109.5
C7—N2—C6	115.9 (2)	H19A—C19—H19B	109.5
C7—N3—C10	122.8 (3)	C16—C19—H19C	109.5
C7—N3—H3A	115 (2)	H19A—C19—H19C	109.5
C10—N3—H3A	121 (2)	H19B—C19—H19C	109.5
C16—N6—C15	124.6 (3)	N4—C10—N3	114.4 (3)
C16—N6—H6	117 (2)	N4—C10—H10A	108.7
C15—N6—H6	118 (2)	N3—C10—H10A	108.7
C11—N5—C15	116.0 (3)	N4—C10—H10B	108.7
C11—N4—C10	123.5 (3)	N3—C10—H10B	108.7
C11—N4—H4A	120 (3)	H10A—C10—H10B	107.6
C10—N4—H4A	117 (3)		
			
C6—N1—C2—C3	−0.1 (5)	C15—N6—C16—C19	176.9 (3)
C6—N1—C2—C1	179.5 (3)	N6—C16—C17—C18	−1.5 (4)
N1—C2—C3—C4	2.1 (5)	C19—C16—C17—C18	179.8 (3)
C1—C2—C3—C4	−177.4 (4)	C16—C17—C18—C14	2.8 (5)
C2—C3—C4—C5	−1.4 (6)	C17—C18—C14—C15	−0.8 (4)
C3—C4—C5—C6	−1.3 (5)	C17—C18—C14—C13	177.1 (3)
C3—C4—C5—C9	177.0 (3)	C11—N5—C15—N6	178.3 (3)
C7—N2—C6—N1	179.2 (3)	C11—N5—C15—C14	−0.7 (4)
C7—N2—C6—C5	0.2 (4)	C16—N6—C15—N5	−175.3 (3)
C2—N1—C6—N2	178.4 (3)	C16—N6—C15—C14	3.8 (4)
C2—N1—C6—C5	−2.5 (5)	C18—C14—C15—N5	176.7 (3)
C4—C5—C6—N2	−177.9 (3)	C13—C14—C15—N5	−1.5 (4)
C9—C5—C6—N2	3.7 (5)	C18—C14—C15—N6	−2.3 (4)
C4—C5—C6—N1	3.1 (4)	C13—C14—C15—N6	179.5 (3)
C9—C5—C6—N1	−175.3 (3)	C15—N5—C11—N4	−176.0 (3)
C6—N2—C7—N3	176.2 (3)	C15—N5—C11—C12	3.0 (4)
C6—N2—C7—C8	−4.9 (4)	C10—N4—C11—N5	−0.9 (5)
C10—N3—C7—N2	−12.6 (4)	C10—N4—C11—C12	−179.9 (3)
C10—N3—C7—C8	168.5 (3)	N5—C11—C12—C13	−2.9 (5)
N2—C7—C8—C9	5.7 (5)	N4—C11—C12—C13	176.0 (3)
N3—C7—C8—C9	−175.5 (3)	C11—C12—C13—C14	0.5 (5)
C7—C8—C9—C5	−1.4 (5)	C18—C14—C13—C12	−176.5 (3)
C4—C5—C9—C8	178.9 (3)	C15—C14—C13—C12	1.5 (4)
C6—C5—C9—C8	−2.8 (4)	C11—N4—C10—N3	74.2 (4)
C15—N6—C16—C17	−1.9 (4)	C7—N3—C10—N4	85.6 (4)

### Hydrogen-bond geometry (Å, °)

**Table:**

*D*—H···*A*	*D*—H	H···*A*	*D*···*A*	*D*—H···*A*
N1—H1···O6^i^	0.88 (4)	1.92	2.794 (4)	168
N3—H3A···O3	0.80 (3)	2.23	2.990 (6)	159
N4—H4A···O5^i^	0.71 (4)	2.56	3.233 (5)	160
N4—H4A···O7^i^	0.71 (4)	2.52	3.133 (5)	145
N6—H6···O1	0.84 (3)	2.00	2.838 (8)	178
C1—H1A···O7^ii^	0.98	2.54	3.501 (3)	167
C1—H1B···O4^iii^	0.98	2.33	3.078 (4)	132
C4—H4···O8^iv^	0.95	2.52	3.392 (7)	152
C10—H10B···O4^iv^	0.99	2.35	3.082 (5)	130
C13—H13···O2^i^	0.95	2.41	3.259 (3)	149
C19—H19B···O5	0.98	2.57	3.351 (6)	136
C19—H19C···O7^v^	0.98	2.58	3.207 (7)	122
C19—H19C···O8^v^	0.98	2.57	3.548 (4)	172

Symmetry codes: (i) −*x*+1, −*y*, −*z*+1; (ii) −*x*+3/2, −*y*, *z*−1/2; (iii) *x*, −*y*+1/2, *z*−1/2; (iv) *x*−1/2, −*y*+1/2, −*z*+1; (v) *x*−1, *y*, *z*.
